The article "Research on the Spatial Agglomeration Characteristics and Influencing Factors of Express Delivery Station Based on DNN" was published in 2022. Journal: Comput Intell Neurosci.

# Research on the Spatial Agglomeration Characteristics and Influencing Factors of Express Delivery Station Based on DNN

**DOI:** 10.1155/2022/3817066

**Published:** 2022-04-22

**Authors:** Zheng Kou

**Affiliations:** College of Business, Yancheng Teachers University, Yancheng 224007, Jiangsu, China

## Abstract

In this paper, the POI data of 736 Cainiao stations in Nanjing is taken as the research sample. With the help of ArcGIS software, the standard deviation ellipse, spatial autocorrelation, average nearest neighbor, cold and hot spot analysis, nuclear density estimation, and other spatial analysis models are used to quantitatively characterize its business mode, spatial distribution characteristics, and equilibrium. Based on DNN, the spatial agglomeration characteristics and distribution directions of the Cainiao station in Nanjing were sorted out, the cold spots and hot spots of the spatial layout were identified, and the spatial differentiation rules and agglomeration patterns were revealed. Finally, the geographically weighted regression analysis model is used to analyze the influencing factors of the spatial agglomeration of the Cainiao station in Nanjing. The research found that Firstly, the proportion of Nanjing Cainiao station operating mode adopting the exclusive mode is 59.1%, the proportion adopting the concurrent operation mode is 33.7%, and the rest adopting the joint operation mode of cooperation with other logistics enterprises. Secondly, Nanjing Cainiao Station gathers in the central city area, forming a “central hot spot.” The urban fringe area does not form a “peripheral cold spot area,” and the whole presents a “1 + 4” five-core agglomeration model across the river. Thirdly, Regional GDP, population density, and the number of convenience stores/supermarkets are the main factors affecting the spatial agglomeration of the Cainiao station in Nanjing.

## 1. Introduction

With the rapid development of e-commerce technology, the variety of online retailers has become increasingly abundant, and the quality has been continuously improved, which has promoted the continuous expansion of the scale of online transactions. In 2021, China's online retail sales amounted to 13088.4 billion yuan, an increase of 14.1% over the previous year. With the rapid development of e-commerce, problems such as insufficient infrastructure facilities, unreasonable layout, and weak service capabilities at the express terminal outlets have become prominent. The “last mile” distribution has become an important bottleneck restricting the development of e-commerce [1]. In order to solve the problem of the last mile of express delivery, European and American countries promoted the self-pickup service through “centralized delivery points” as early as 2001 [2]. In Singapore and Japan, second-generation self-service kiosks and “convenience store pickup mode” [3] have also appeared. Alibaba followed the example of foreign self-pickup spaces and teamed up with major private express companies such as SF Express and “Four Links and One Delivery” to create “cainiaoPosts.” China Post Group has also set up self-pickup services in their respective outlets [4], and technology companies such as Fengchao and China Post Express have successively launched smart express cabinets. The location and layout of these terminal distribution facilities are jointly restricted by many factors such as population density [5], transportation cost [6], land use type, business district scale [7], transportation facilities [8], and other factors, showing different distribution patterns and agglomeration characteristics. So is the distribution of rookies in the city discrete or agglomerated? What factors affect the appearance of this state? What is the extent of its impact? These problems will become the key to cracking the unreasonable layout of express delivery infrastructure and solving the “last mile” distribution problem.

In recent years, research-based on big data has increased day by day, innovating research methods and enriching research fields. Point of Interest (POI) is a kind of point-like data representing real geographic entities, usually with rich semantic features and spatiotemporal dynamic correlation characteristics. It is widely used in urban transportation network settings [9, 10], urban spatial structure analysis [11, 12], urban public cultural facilities service level spatial distribution pattern and difference analysis [13–15], residents' daily activities [16, 17], etc. Recently, it has also been used to study the field of express delivery infrastructure layout [18], but the research on the spatial layout of the Cainiao station based on POI data is still insufficient.

Existing studies mostly discussed the distribution characteristics of express self-pickup points such as Cainiao Station and put forward several suggestions on the layout of express terminal facilities but failed to reveal the deep-seated reasons and mechanisms affecting this distribution, and the research conclusions have limitations. Based on this, based on the perspective of geography, this article uses the POI data of 736 Cainiao stations in Nanjing as a research sample to try to reveal the spatial layout and agglomeration mode of the Cainiao stations. And explore the in-depth mechanism that affects this layout and provide a reference for the equal and balanced configuration of express facilities at the end of the city.

## 2. Research Area, Methods, and Data Sources

### 2.1. Overview of the Study Area

Located in the lower reaches of the Yangtze River, Nanjing is an important industrial city and economic center city in the country and an important transportation hub and logistics node city in East China. There are 11 districts in Nanjing, namely Xuanwu District, Gulou District, Qinhuai District, Yuhuatai District, Jianye District, Pukou District, Qixia District, Jiangning District, Lishui District, Liuhe District, and Gaochun District. The total area is 6587 km^2^, with a permanent population of 9.42 million at the end of 2021. As the capital of Jiangsu Province and the central city of the Yangtze River Delta, Nanjing has a developed economy, dense colleges, and a relatively concentrated population, which has a great demand for express delivery stations. According to the data: In 2021, the total retail sales of consumer goods in Nanjing will be 789.941 billion yuan. The proportion of online retail sales in commodity retail sales reached 22.4%, an increase of 4.0 percentage points over the previous year. During the Double Eleven period, the express business volume reached 107.04 million pieces.

### 2.2. Research Methods

#### 2.2.1. Standard Deviation Ellipse Model

Standard Deviational Ellipse (SDE) is a measurement analysis method proposed by D.Welty Lefever [19] to measure the direction and distribution of a set of data, which can be used to judge the distribution direction characteristics of a data set. The semimajor axis of the ellipse represents the main distribution direction of the data in space, and the semiminor axis represents the distribution range of the data in space. The greater the difference between the long and short semiaxes (the greater the flatness), the more obvious the directionality of the data set [20]. The calculation formula is as follows:

(1) $$\begin{array}{c} SED_{x}=\sqrt{\frac{{\sum_{i=1}^{n}\left(x_{i}-\bar{x}\right)}^{2}}{n}},\\ SED_{y}=\sqrt{\frac{{\sum_{i=1}^{n}\left(y_{i}-\bar{y}\right)}^{2}}{n}}. \end{array}$$

In the formula, *x*_*i*_ and *y*_*i*_ are the spatial position coordinates of a feature, $\left\{\bar{x}|\bar{y}\right\}$ represents the average center of the feature, and *n* represents the total number of features.

#### 2.2.2. Spatial Autocorrelation Analysis

Spatial autocorrelation is mainly used to test a certain geographic phenomenon or the overall distribution of a certain attribute value and judge whether the geographic phenomenon or attribute value has agglomeration characteristics in space [21]. In view of the different spatial scope of the research, the measure of spatial autocorrelation can be divided into global spatial autocorrelation and local spatial autocorrelation [22]. This paper uses global spatial autocorrelation to measure whether the spatial layout of the Cainiao station in Nanjing has agglomeration characteristics. The global spatial autocorrelation index is called Global Moran's I, and its calculation formula is as follows:

(2) $$\begin{array}{c} I=\frac{n\sum_{i=1}^{n}\sum_{j=1}^{n}wij\left(y_{i}-\bar{y}\right)\left(y_{j}-\bar{y}\right)}{\left(\sum_{i=1}^{n}\sum_{j=1}^{n}w_{ij}\right)\sum_{i=1}^{n}{\left(y_{j}-\bar{y}\right)}^{2}}. \end{array}$$

In the formula, I is the local spatial autocorrelation index, *n* represents the number of spatial units, *y*_*i*_ and *y*_*j*_ represent the attribute values of spatial units *i* and *j*, respectively, and *w*_*ij*_ represents the proximity relationship between regions *i* and *j*.

The value range of Moran's I index is [−1, 1]. When Moran's I > 0, it means positive correlation; when Moran's I = 0, it means no correlation; when Moran's I < 0, it means negative correlation. The closer the value of Moran's I index is to 1, the smaller the overall spatial disparity, and the closer the value of Moran's I index is to −1, the greater the overall spatial disparity.

#### 2.2.3. Kernel Density Estimation Method

The kernel density analysis method was proposed by Rosenblatt (1955) and Emanuel Parzen (1962). This method is used to calculate the density of elements in their surrounding fields and to explore the probability of point elements occurring in different geographic spatial locations within a region. The higher the nuclear density value, the higher the probability of event occurrence and the denser the points [23]. The calculation formula is as follows:

(3) $$\begin{array}{c} f_{h}\left(x\right)=\frac{1}{nh}\sum_{i=1}^{n}\left(\frac{x-x_{i}}{h}\right). \end{array}$$

In the formula: *f*_*h*_(*x*) is the kernel function, (*x* − *x*_*i*_)  represents the distance from *x* to *x*_*i*_, *h* > 0 is the width, and the larger the value of *f*_*h*_(*x*), the denser the distribution.

#### 2.2.4. Average Nearest Neighbor Index

The average nearest neighbor index is mainly used to determine the overall spatial agglomeration characteristics of elements, and the average nearest neighbor tool is used to measure the distance between the centroid of each element and its neighbors. Then the average of these nearest neighbor distances can be obtained to get the nearest neighbor index (ANN) [24]. If ANN<1, it means that the spatial distribution of the sample is a clustering pattern; if ANN>1, it means that the spatial distribution pattern of the sample tends to spread. The calculation formula is as follows:

(4) $$\begin{array}{c} \text{ANN}=\frac{\bar{D_{O}}}{\bar{D_{E}}}=\frac{1/n\sum_{i=1}^{n}d_{i}}{0.5*\sqrt{A/n}}. \end{array}$$

In the formula: $\bar{D}o$ is the average distance between the measured element and its nearest neighbor, and $\bar{D}$*E* is the average expected distance between the elements in the random mode. *d*_*i*_ is the distance between element *i* and its nearest neighbors, *n* is the number of regional elements, and A is the area of the study area.

#### 2.2.5. Geographically Weighted Regression Model (GWR)

The geographically weighted regression model introduces the spatial location of the data into the linear regression model to explore the spatial nonstationarity of geographic data. Embed the spatial position of the sample data into the regression equation. The expression is as follows:

(5) $$\begin{array}{c} Y_{i}=\partial_{0}\left(u_{i},v_{i}\right)+\sum_{n=1}^{i}\partial_{i}\left(u_{i},v_{i}\right)\lambda_{i}+\varepsilon_{i}. \end{array}$$

In the formula, *Y*_*i*_ is the number of rookies in the dependent variable, and ∂_*i*_(*u*_*i*_, *v*_*i*_) is the independent variable with the space centroid. ∂_*o*_(*u*_*i*_, *v*_*i*_ ) is a constant term with space centroid, *λ*_*i*_ is the regression coefficient, and *ε*_*i*_ is a random error term.

#### 2.2.6. Deep Neural Networks (DNN)

DNN is sometimes called a multilayer perceptron. According to the location of different layers in DNN, the neural network layer inside DNN can be divided into three categories: input layer, hidden layer, and output layer, as shown in Figure 1.

In Figure 1, layers are fully connected; that is, any neuron in *i*-th layer must be connected with any neuron in the (*i*+1)-th layer. Although DNN looks very complex, the small local model is the same as the perceptron, that is, a linear relationship *f*=∑*w*_*i*_*x*_*i*_+*b* plus an activation function *σ*(*f*).

Assuming that the selected activation function is *σ*(*f*) and the output value of the hidden layer and the output layer is *α*, for the three-layer DNN shown in Figure 2, using the same idea as the perceptron, we can use the output of the previous layer to calculate the output of the next layer, that is, the so-called DNN forward propagation algorithm.

For the output *α*_1_^2^,  *α*_2_^2^,  *α*_3_^2^ of the second layer,

(6) $$\begin{array}{c} \alpha_{1}^{2}=\sigma \left(f_{1}^{2}\right)=\sigma \left(w_{11}^{2}x_{1}+w_{12}^{2}x_{2}+w_{13}^{2}x_{3}+b_{1}^{2}\right),\\ \alpha_{2}^{2}=\sigma \left(f_{2}^{2}\right)=\sigma \left(w_{21}^{2}x_{1}+w_{22}^{2}x_{2}+w_{23}^{2}x_{3}+b_{2}^{2}\right),\\ \alpha_{3}^{2}=\sigma \left(f_{3}^{2}\right)=\sigma \left(w_{31}^{2}x_{1}+w_{32}^{2}x_{2}+w_{33}^{2}x_{3}+b_{3}^{2}\right). \end{array}$$

Using the matrix method, the output of *i*-th layer can be expressed as follows:

(7) $$\begin{array}{c} \alpha^{i}=\sigma \left(f^{i}\right)=\sigma \left(W^{i}\alpha^{i-1}+b^{i}\right). \end{array}$$

DNN forward propagation algorithm is to use several weight coefficient matrices *W* and bias vector *b* to carry out a series of linear operations and activation operations with the input value vector *x*, starting from the input layer, calculating backward layer by layer until the operation reaches the output layer, and the output result is the value.

For *W* and *b*, the concept of the cost function is introduced. The cost function is used to adjust the parameters to make the model approach the real event model. It is defined as follows:

(8) $$\begin{array}{c} C\left(w,b\right)=\frac{1}{2n}{\sum_{x}\left\|y\left(x\right)-\alpha \right\|}^{2}, \end{array}$$

where *n* is the number of samples, *y* corresponds to the correct result of the sample, and *α* is the result of DNN under the current sample input.

### 2.3. Data Source

With the advancement of positioning technology and the development of mobile Internet, map positioning and location-based services (LBS) are widely used in the Internet economy, and spatial geographic data represented by POI has been continuously enriched and improved [25]. This article uses the “POI query” function provided by “Maice Data MDT” as the data source and enters the keywords “Nanjing + Cainiao Station”, “Nanjing + China Post,” and “Nanjing + convenience store/supermarket.” After data sorting and elimination, coordinate correction processing, and geographic information correction and completion processing, 736 POI data from Nanjing Cainiao Station, 248 POI data from postal sites, and 1,630 POI data of convenience stores/supermarkets were obtained (as of April 2020). In addition to the POI data, the land area, population, and regional GDP of the municipal districts of Nanjing are derived from the “Nanjing Statistical Yearbook 2019.” The administrative map of Nanjing is divided into 80 small areas according to streets, towns, and districts, using the spatial connection tools in ArcGIS. The POI data of Cainiao Station, Convenience Store/Supermarket, and Post Station were spatially connected with the divided administrative area map of Nanjing City, and the number of Cainiao Station, Convenience Store/Supermarket, and Post Station in 80 districts was obtained. And through the survey of the relevant socioeconomic conditions of the streets, towns, and districts, the data of the regional GDP, population, and the number of communities under its jurisdiction are obtained (Table 1).

## 3. Analysis of Agglomeration Characteristics of the Cainiao Station in Nanjing

### 3.1. Analysis of Basic Characteristics

#### 3.1.1. Relying on Form Characteristics

According to the data analysis of different types of business locations of Cainiao Station outlets by DNN, they are divided into three types: franchise, concurrent, and joint operation. The specific division is shown in Table 2.

By combing through the POI data of 736 Cainiao stations in Nanjing, we found that there are 435 post outlets with independent business premises in the franchise model, accounting for 59.1%. There are 248 Cainiao Station outlets under the concurrent operation model, accounting for 33.7%. In the part-time operation model, the proportion of operations that rely on supermarkets and convenience stores is as high as 48.6%, followed by fruit stores and hardware stores. By relying on these commercial facilities, it can not only provide convenient express delivery services for nearby residents but also attract a certain amount of passenger flow for commercial facilities. The remaining 53 Cainiao Station outlets and other logistics companies' express outlets shared their business premises using a joint operation model (Figure 3). The difference in reliance is not only directly related to the business volume of self-pickup points but also affected by the business strategy of the shopkeeper.

#### 3.1.2. Service Object Characteristics

The setting of express delivery points aims to improve the efficiency of the “last mile” of logistics so as to facilitate the self-pickup of residents. Therefore, express delivery points are usually located near the entrances and exits of people in the community and in dense areas of commercial business activities. According to the service objects of Nanjing Cainiao Station, it can be seen that the service objects of Nanjing Cainiao Station are mostly communities (77.27%), commercial intensive areas (11.82%), and universities (8.18%). There are fewer layouts in areas such as industrial parks, villages and towns, and scenic spots（Table 3. This is mainly due to the overall cost and benefit of the Cainiao Station site selection, so most of the sites are located in central urban communities with a large number of parcels and commercial streets and universities in other parcel-intensive areas, and they rarely extend to urban fringe areas.

#### 3.1.3. Service Distance Characteristics

The setting of the express delivery point is mainly to relieve the distribution pressure caused by the rapid increase in the volume of express parcels and to solve the contradiction between the mismatch between express delivery time and customer pickup time. Service distance affects the time value that consumers need to pay for extraction, and a reasonable layout is critical to improving the consumer's shopping experience. By analyzing the distance between the Cainiao station in Nanjing and the entrance and exit of the service object (Figure 4), it can be seen that as the distance from the entrance and exit of the community increases, the number of the Cainiao station shows a law of “increasing first and then decreasing.” And the number of Cainiao Posts within 100–150 meters from the entrance and exit is the largest, and the number of Cainiao Posts more than 400 meters from the entrance and exit is less. Judging from the cumulative percentage, 86.55% of the Cainiao stations in Nanjing have a service distance of 200 m. Based on a person's walking speed of 4-5 km/h, 95.65% of the Cainiao stations are within 5 minutes of walking.

### 3.2. Analysis of Spatial Distribution Characteristics

#### 3.2.1. Quantity Distribution Characteristics

Using ArcGIS spatial join tool (spatial join) to obtain the POI point data of the Cainiao station and the data of the districts of Nanjing City, it can be seen after spatial aggregation statistical analysis (Figure 5). Nanjing Cainiao Station is mainly concentrated in 5 main urban areas and 3 main urban subcentral areas. There are a total of 665 Cainiao stations in these eight urban areas, accounting for 90.35% of the city's Cainiao stations. Among them, the ratio of Cainiao stations in Qixia District, Jiangning District, and Pukou District ranks in the top 4, with an average of 2.01, 1.64, and 1.31 Cainiao stations per 10,000 people, respectively. The reason is that these three main cities and subcenters have three university cities: Xianlin, Jiangning, and Pukou. The concentration of universities has stimulated the demand for e-commerce shopping, which has driven the growth of Cainiao's outlets. It is worth noting that the population density of the Gulou District in the main urban area is as high as 17,437 people/km2, but the number of Cainiao posts per 10,000 people is only 0.82.

#### 3.2.2. Spatial Distribution Characteristics

The POI data layer of Nanjing Cainiao Station was superimposed on the administrative division map of Nanjing City by ArcGIS software, and the spatial distribution map of Nanjing Cainiao Station was obtained (Figure 6(a)). At the same time, use the “Direction Distribution” tool to obtain the standard deviation ellipse analysis chart of the Cainiao station in each city (Figure 6(b)). According to Figure 4, the layout of the Cainiao station in Nanjing presents the following characteristics.

1. The spatial layout is unbalanced, showing the characteristics of “more in the north and less in the south, dense in the middle and sparse in the periphery.”
2. The layout of the Cainiao station in Nanjing is concentrated in the north-central part and rarely in the Lishui District and Gaochun District in the south. Specifically, it is mainly concentrated in and around the densely populated main urban area near the Yangtze River Basin, with few surrounding districts and counties. The reason is that the main urban area is the political, economic, and cultural center of the city, and the construction of urban supporting facilities is relatively complete. It brings together the city's commercial centers, residential centers, and college areas to drive a large amount of self-provisioning demand.
3. The distribution direction is consistent with the shape of the city, pointing to the “southeast-northwest” direction
4. The standard deviation ellipse analysis chart of Nanjing Cainiao Station (Figure 6(b)) shows that the distribution of Cainiao Station is roughly along the “southeast-northwest” direction and the difference between the long and short semiaxes is large, and the directionality is obvious. It is consistent with the administrative division, regional development level, and population distribution of Nanjing. The number and distribution density of the Cainiao stations in the ellipse are higher than those outside the circle, which is consistent with the characteristics of “dense in the middle and sparse in the periphery.”
5. Coinciding with residential land and scarcer quantitative distribution of marginal settlements

The express delivery site itself exists to serve urban residents, so it is closely adjacent to the distribution of residential areas. The land-use types where the self-pickup sites are located are mostly residential land, but there are still a considerable number of residential areas without self-pickup sites. It can be seen from Figure 6 that almost all the residential land in the central urban area is distributed with Cainiao Stations. However, in the northern part of Liuhe District, the southern part of Nanjing Lishui District, and the Yuancheng District in the surrounding area of Gaochun District, there are fewer Cainiao Stations. As urbanization develops and the distribution of residents increases, these areas will become new expansion areas.

### 3.3. Analysis of Spatial Agglomeration Characteristics

#### 3.3.1. Spatial Autocorrelation Analysis and Average Nearest Neighbor Analysis

*(1)Spatial Autocorrelation Analysis.* In order to make the calculation results more accurate, first use the “Calculate the distance between neighbors” tool to calculate the “maximum distance” (14381 m in this article) and set this distance as the distance threshold specified in “Spatial Autocorrelation Analysis” and “Hot Spot Analysis.” Ensure that each feature in the input feature class has at least N adjacent points.

According to the calculation result of the global autocorrelation coefficient, Moran's I (Figure 7(a)), it can be seen that the autocorrelation coefficient Moran's I > 0 of the Cainiao station in Nanjing, indicating that there is a positive correlation in the spatial distribution of the Cainiao station in Nanjing. *P* < 0.1; that is, the probability that the spatial distribution of the Cainiao station in Nanjing is less than 10% is random, and the probability that the Cainiao has gathered in Nanjing is greater than the probability of random distribution and can significantly reject the null hypothesis; the result is credible.

*(2) Average Nearest Neighbor Analysis.* Input the point map data into the “Average Nearest Neighbor” tool and calculate the average observation distance, expected average distance, and nearest neighbor index of Nanjing Cainiao Station to be 638.52 m and 1464.55 m, respectively. The average nearest neighbor index ANN is 0.4360, ANN<1, indicating that the Cainiao station is clustered in Nanjing.

#### 3.3.2. Hot Spot Analysis and Nuclear Density Analysis

*(1)Hot Spot Analysis (Getis-Ord Gi).* The hot spots (high-value agglomeration areas) of Nanjing Cainiao Inn outlets are concentrated in the central city. Specifically (Figure 8(a)), they are mainly distributed in the central city streets of the five main city areas and three main city subcity areas. For example, Yanziji Street, Yaohua Street, and Baguazhou Town in Qixia District; Taishan Street and Yanjiang Street in Pukou District; Shangfang Town and Qilin Town in Jiangning District. The Nanjing Economic and Technological Development Zone and Qixia Street in Qixia District, Dingshan Street in Pukou District, Tiexinqiao Street in Yuhuatai District, and Chunhua Town in Jiangning District all have subhot spots. However, there is no cold spot area (low-value agglomeration area), indicating that Nanjing Cainiao Station has developed traffic, densely populated, and widespread communities, forming a “central hot spot.” The reason is that the central urban area has become the main hot spot due to the great demand for express delivery points due to the developed traffic, dense population, and wide distribution of communities. The formation of cold spots is due to the distance from the city center, the lack of traffic, and the sparse population. Considering costs and benefits, companies generally set up Cainiao stations in areas where residents and universities are concentrated.

*(2) Nuclear Density Analysis.* Based on the agglomeration space obtained by the hot spot analysis, the “nuclear density analysis” tool in ArcGIS is used to analyze the agglomeration mode of the Cainiao station in Nanjing. When analyzing, set the output pixel size of the nuclear density analysis to 150 m *∗* 150 m, and the search radius to 2000 m. It can be seen from Figure 8(b) that Nanjing Cainiao Station presents a “multicore agglomeration mode” in the central urban area and subcentral urban areas of the main city, forming a small agglomeration phenomenon in outlying suburban counties. Its agglomeration mode is specifically expressed as the “Gejiang ‘1 + 4' Penta-core agglomeration mode: In the north of the Yangtze River and Pukou, Yanjiang Street and Taishan Street form a core area of agglomeration. In the Gulou District to the south of the Yangtze River, Baixia District in Qinhuai District, and Shangfang Town and Shangyuan Street in Jiangning District, Qilin Town has formed four high-gathering core areas. Yanziji Street, Xuanwu District, and Yuhuatai District in Liuhe District and Qixia District form secondary core areas. Except for the small high-density agglomeration core area of Qilin Town, the remaining four high-density agglomeration core areas are connected in a line and distributed along the “southeast-northwest.”

## 4. Research on the Influencing Factors of the Spatial Agglomeration of the Rookies in Nanjing

### 4.1. Variable Selection and Description

The existence of geographical things has its own special selection characteristics. Reasonable layout and efficient agglomeration are conducive to resource sharing and mutual cooperation in order to achieve the purpose of saving costs and improving efficiency. Chen Lulu (2019) proposed in the study that the number of Cainiao Station sites is affected by factors such as land area, total population, population density, number of subdistrict offices, and regional GDP. JI Qin et al. (2021) [26]proposed in their research that the layout of self-pickup points is affected by factors such as economy, population, land use type, and traffic. Through the above research on the basic characteristics and spatial agglomeration characteristics of the Cainiao station in Nanjing, combined with the research and analysis of relevant theoretical literature, this paper takes the macroscopic aspect of the land area, regional GDP, year-end population, population density, and microscopic aspects of the number of convenience stores/supermarkets, communities, and postal sites as independent variables. Take the number of Cainiao posts as the explained variable and conduct an empirical analysis. The selection of specific variables is shown in Table 4:

### 4.2. Analysis of Research Results

#### 4.2.1. Correlation Coefficient Analysis

Use spass22.6 software to analyze the Pearson correlation coefficient between the number of Cainiao posts in Nanjing and the area of land, regional GDP, population, population density, convenience stores/supermarkets, communities, China Post, and Fengchao cabinets. According to the research results (Table 5), the number of Cainiao posts is negatively correlated with the area of land under its jurisdiction; it has a strong correlation with the area's gross product, year-end population, population density, the number of convenience stores/supermarkets, and the number of communities; it has a strong correlation with the number of postal sites. There is a certain correlation between these influencing factors, and then the influencing factors with collinearity are eliminated in the multiple regression model.

#### 4.2.2. Multiple Linear Regression Analysis

In this study, the number of Cainiao posts in Nanjing is used as the explanatory variable, and the land area under its jurisdiction, regional GDP, year-end population, population density, number of convenience stores/supermarkets, number of communities, and number of postal stations are used as explanatory variables of dependent variables. Establish a multiple linear regression model. The regression equation is as follows:

(9) $$\begin{array}{c} Y_{i}=C+\beta_{1}X_{1}+\beta_{2}X_{2}\cdots +\beta_{i}X_{i}. \end{array}$$

In the formula, *y*_*i*_ represents the explained variable of the i-th area, *x*_*i*_ represents the explanatory variable, C is the constant term, and *β*_*i*_ is the regression coefficient.

According to the analysis result of the multiple linear regression model, R2 is 0.922（Table 6. It means that the area of land under its jurisdiction, the regional GDP, the population at the end of the year, the population density, the number of convenience stores/supermarkets, the number of communities, and the number of postal stations are the reasons that affect 92.2% of the number of Cainiao Posts. From the standard coefficient and Sig value, it can be seen that the regional GDP, population density, number of convenience stores/supermarkets in the model are positively correlated with the spatial layout of the Cainiao station. That is to say, the higher the regional GDP, the greater the population density, and the more convenience stores/supermarkets, the more concentrated the layout of the Cainiao Station. However, the area under its jurisdiction, the number of population, the number of communities, the number of postal stations, and the layout of the Cainiao post are not significantly affected, so they are eliminated.

#### 4.2.3. Geographically Weighted Regression Model Analysis (GWR Model)

In order to further study the factors affecting the distribution of the number of Cainiao stations in Nanjing and to visualize the factors, based on the regression analysis, this study introduces a geographically weighted regression model to modify and improve the original model. The R2 of the geographically weighted regression model is 0.939598, which is greater than 0.921（Table 7). It can be seen that the fit of the model is better than the multiple linear regression model.

According to Figure 9, the regression coefficient of regional GDP is between 0.21622 and 0.23433, and the regression coefficient is positive. It shows that regions with a high level of regional economic development will stimulate more production and living logistics needs and generate a large amount of demand for self-pickup packages. Cainiao Posts will also be concentrated in areas with a high regional GDP. The higher the regional GDP, the greater the number of Cainiao Posts distributed. The regional GDP of the jurisdiction where the five high-density agglomeration core areas are located accounts for 72.36% of the city's GDP. The regression coefficient in the north of the regional GDP in the figure is higher than the regression coefficient in the south, showing a phenomenon of north-south differentiation, which is also consistent with the spatial distribution characteristics of Cainiao Station. The regression coefficient of population density is between 0.00104 and 0.001236, and the regression coefficient is positive, indicating that the higher the population density, the denser the layout of the Cainiao post. The distribution of the neighbors of the Cainiao station is highly dependent on the population. The Cainiao station and the population distribution are obviously convergent, and the agglomeration of the two is complimentary. Therefore, the agglomeration of a certain scale of the population is a necessary condition for the agglomeration of rookies. The regression coefficient of the number of convenience stores/supermarkets is between 0.158000 and 0.164000, and the regression coefficient is positive. It shows that the more convenience stores/supermarkets, the more obvious the agglomeration of Cainiao stations. Convenience stores/supermarkets are the commercial service facilities most relied on by Cainiao Inns, and their development time is relatively long and mature. Therefore, their layout conditions directly affect the concentration or dispersion of Cainiao Inns.

## 5. Conclusion and Discussion

### 5.1. Main Conclusion

This study uses ArcGIS software to quantify its spatial distribution characteristics and equilibrium using spatial analysis models such as standard deviation ellipse, spatial autocorrelation, average nearest neighbor, cold hot and hot spot analysis, and nuclear density estimation. On this basis, the management mode and spatial layout characteristics of the Cainiao station in Nanjing are sorted out, the cold spots and hot spots of the spatial layout are identified, and its spatial differentiation law and agglomeration mode are revealed. Finally, the geographically weighted regression analysis model (GWR model) is used to analyze the factors affecting the spatial agglomeration of the Cainiao station in Nanjing. The main research conclusions are as follows:

- In the business model of Nanjing Cainiao Station, 59.1% use the exclusive mode, 33.7% use the concurrent mode, and the rest use the joint operation mode of cooperation with other logistics companies' distribution points. In the concurrent mode, Cainiao Inn mostly relies on supermarkets, convenience stores, fruit shops, and other public service facilities. From the perspective of the service targets of Cainiao Inn, it mainly serves communities, commercial streets, and university districts, followed by industrial parks, villages and towns, and scenic spots. The distance between the Cainiao station and the service object exhibits the law of “increasing first and then decreasing”. 95.65% of the Cainiao station is located within 300 meters from the entrance and exit of the community, within a 5-minute walk.
- Nanjing Cainiao Stations are mainly distributed in 5 main urban areas and 3 main urban subcentral areas, and their spatial distribution presents the characteristics of “more in the north and less in the south, dense in the middle and sparse in the periphery.” The distribution direction is consistent with the shape of the city, pointing to the “southeast-northwest” direction. From the perspective of agglomeration characteristics, agglomeration in the city's central urban area forms a “central hotspot area” and secondary hotspot areas are formed outside the hotspots of the three main city subcentral urban areas. There is no “peripheral cold spot” in the urban fringe, and the agglomeration mode is the “Gejiang “1 + 4” penta-nucleus agglomeration mode.”
- Regional GDP, population density, and the number of convenience stores/supermarkets are the main factors that affect the spatial agglomeration of the Cainiao station. The agglomeration of a certain scale of the population is a necessary condition for the agglomeration of the Cainiao station. Regions with a high level of regional economic development will stimulate more production and living logistics needs and generate a large amount of demand for self-pickup packages. Convenience stores/supermarkets are the commercial service facilities most relied on by Cainiao Inns, and their development time is relatively long and mature. Their layout conditions directly affect the concentration or dispersion of Cainiao Inns.

## 6. Discussion

Based on the spatial distribution characteristics of the Cainiao station in Nanjing and the differences in various regions, this article puts forward the following development suggestions: ① The layout of the Cainiao station is combined with the development planning of each administrative district. In the planning and construction of Cainiao Station, the functional structure of each administrative area should be fully considered, combined with factors such as the population, area, and economic development level of the jurisdiction, and key layouts in residential areas with a large flow of people and limited urban space, commercial vitality points, and colleges and universities. For various parks with a great demand for parcels, it is also necessary to set up Cainiao Station. Through a map survey of the industrial/industrial parks in different jurisdictions of Nanjing, it is found that these parks have logistics companies. Therefore, in industrial/industrial parks where there is no Cainiao station, a joint venture model of cooperation with park logistics companies can be used to serve the park staff. ②When considering the layout of the Cainiao station, it is necessary to consider whether it is consistent with the layout plan of other public service facilities such as postal stations and Fengchao self-pickup cabinets to avoid repeated construction. Public service facilities have a large investment in construction, and their operation and maintenance costs are high as public welfare facilities, so it is very necessary to ensure the effective use efficiency of the facilities after they are completed. However, due to the early construction of some communities and the relatively concentrated communities, the surrounding land resources are relatively tight. In order to save urban space, cooperation with other public service facilities in the city should be considered. ③The construction of the Cainiao station must fully consider the distance from the entrance and exit of the community and follow the principle of facilitating the residents' self-report behavior. The current mode of transportation for residents to pick up express delivery is mainly on foot, and the travel distance is limited. Therefore, a pickup radius of 250–500 m from the express delivery point is good. In the future, the spatial layout of express delivery points should fully consider the walking distance and convenience of residents. Parking lots and bus traffic stations with a large flow of people should also be used as important areas for the future planning and layout of express delivery points.

This article systematically sorts out the operation mode, spatial distribution, and agglomeration characteristics of Nanjing Cainiao Station and reveals its spatial distribution characteristics and agglomeration mode. However, due to limited research data, research on the layout of Cainiao stations in other cities needs further attention in the future. In addition, in future research, postal sites and self-pickup counters with the same function can be selected for horizontal comparison, and the self-pickup behavior of urban residents can be deeply discussed and studied.

## Figures and Tables

**Figure 1:** The structure of DNNs.

**Figure 2:** DNN forward propagation algorithm.

**Figure 3:** Types of Cainiao station in Nanjing city.

**Figure 4:** Service distance of Cainiao station in Nanjing city.

**Figure 5:** Spatial distribution of the Cainiao station in Nanjing city.

**Figure 6:** The spatial distribution and standard deviation ellipse analysis diagram of the Cainiao station in Nanjing (a). Spatial distribution of the Cainiao station (b). Standard deviation ellipse analysis chart.

**Figure 7:** Spatial autocorrelation analysis and average nearest neighbor analysis of the Cainiao station in Nanjing (a). Spatial autocorrelation analysis graph (b). Average nearest neighbor analysis graph.

**Figure 8:** Hot spot analysis and nuclear density analysis diagram of Cainiao Station in Nanjing (a). Hot spot analysis (b) Nuclear density analysis chart.

**Figure 9:** Regression coefficient distribution.

**Table 1:** Number of Cainiao posts and socioeconomic conditions in each district of Nanjing.

Area type	City area	Area/km^2^	GDP (100 million yuan)	Population/person	The population density (People/km^2^)	Number of convenience stores (a)	Number of cells (a)	Number of postal sites (a)	Number of cainiao stations (a)
Main city	Xuanwu district	75.46	895.37	473210	6271	122	632	33	53
	Qinhuai district	49.11	1043.03	690555	14061	121	1014	24	80
	Gulou district	53.00	1478.37	924180	17437	84	1384	24	76
	Jianye district	82.93	746.87	378932	4569	68	424	5	25
	Yuhuatai district	132.39	651.05	297850	2250	105	364	16	47
Main city and subcity	Qixia district	395.44	1394.62	512448	1296	170	488	23	103
	Jiangning district	1563.32	2163.60	1123270	719	415	939	44	184
	Pukou district	698.15	1050.11	743182	1065	189	509	25	97
Other urban areas	Liuhe district	1295.27	1227.90	932669	720	273	470	25	49
	Lishui district	1063.67	789.09	443821	417	59	250	15	21
	Gaochun district	790.23	682.59	449288	569	24	273	14	1
Citywide		6198.97	12122.60	6969405	1124	1630	6747	248	736

**Table 2:** The division of Nanjing Cainiao Station by type.

Business model	Basis of division
Franchise	The outlets of Cainiao yizhan with independent business premises
Concurrent	Relying on other public service facilities business premises (supermarkets, convenience stores, fruit stores, beauty salons, hardware stores, mobile communication stores, property centers, etc.)
Joint operation	Share business premises with other logistics enterprise units.

**Table 3:** Service targets of Cainiao station in Nanjing city.

Service object type	Amount	Ratio （%）
Community	568	77.27
Commercial street	87	11.82
Colleges	60	8.18
Industrial park	14	1.91
Town	5	0.68
Scenic spot	2	0.27

**Table 4:** Spatial agglomeration factors of Cainiao station in Nanjing city.

Variable		Description
Macro	Area under jurisdiction	The area of land under its jurisdiction provides a guarantee for the expansion of urban space. The larger the area under its jurisdiction, there are often more Cainiao posts.
	GDP	Areas with high regional GDP indicate that the better the level of economic development, they tend to attract population and capital agglomeration, and the demand for Cainiao posts will gradually increase.
	Total population at the end of the year	An area with a larger population means that the more demand for e-commerce infrastructure, the more the layout of the Cainiao station.
	The population density	High-density crowded areas will have a large amount of package demand, which in theory will drive the increase in the number of Ccainiao posts.
Micro	Number of convenience stores/supermarkets	The number of convenience stores/supermarkets provides support for Cainiao station, and the agglomeration and dispersion of convenience stores/supermarkets affect the aggregation and dispersion of Cainiao station.
	Number of communities in jurisdiction	The number of communities directly reflects the size of the population. The greater the number of communities in the jurisdiction, the greater the demand for Cainiao station.
	China post office	Cainiao post and postal outlets have complementary functions. Generally, the more postal outlets, the fewer the number of Cainiao post.

**Table 5:** Correlation analysis.

	Number of Cainiao stations	Land area	GDP	Population at the end of the year	The population density	Number of convenience stores/supermarkets	Number of cells	Number of postal sites
Number of Cainiao stations	1							
Land area	−0.236 ^*∗*^	1						
GDP	0.928 ^*∗*^ ^*∗*^	−0.197	1					
Population at the end of the year	0.900 ^*∗*^ ^*∗*^	−0.166	0.984 ^*∗*^ ^*∗*^	1				
The population density	0.830 ^*∗*^ ^*∗*^	−0.364 ^*∗*^ ^*∗*^	0.878 ^*∗*^ ^*∗*^	0.987 ^*∗*^ ^*∗*^	1			
Number of convenience stores/supermarkets	0.940 ^*∗*^ ^*∗*^	−0.131	0.861 ^*∗*^ ^*∗*^	0.835 ^*∗*^ ^*∗*^	0.693	1		
Number of cells	0.836 ^*∗*^ ^*∗*^	−0.262 ^*∗*^	0.933 ^*∗*^ ^*∗*^	0.946 ^*∗*^ ^*∗*^	0.920 ^*∗*^ ^*∗*^	0.691	1	
Number of postal sites	0.779 ^*∗*^	−.100	.853 ^*∗*^ ^*∗*^	0.841 ^*∗*^ ^*∗*^	0.711 ^*∗*^	0.765 ^*∗*^	0.827 ^*∗*^ ^*∗*^	1

^*∗*^. Significantly correlated at the 0.05 level (two-sided);  ^*∗*^ ^*∗*^. Significantly correlated at the 0.01 level (two-sided).

**Table 6:** Multiple linear regression analysis results.

Model	Nonstandardized coefficient		t	Sig
	B	Standard error		
(Constant)	−1.087	1.481	−0.734	0.465
Land area	0.001	0.016	0.059	0.953
GDP	0.047	0.015	3.161	0.002 ^*∗*^ ^*∗*^
Population at the end of the year	−6.582	0.000	−2.520	0.118
The population density	0.001	0.001	1.584	0.014 ^*∗*^
Number of convenience stores/supermarkets	0.319	0.052	6.096	0.000 ^*∗*^ ^*∗*^
Number of communities	0.025	0.015	1.744	0.085
Number of postal sites	−0.037	0.240	−1.547	0.126

^*∗∗*^＜0.01;  ^*∗*^＜0.05; *R*2 = 0.922.

**Table 7:** GWR model results.

Index	Result
EffectiveNumber	11.788726
Sigma	4.297719
AICc	477.793169
*R* ^2^	0.939598
R^2^Adjusted	0.930183

## Data Availability

The data used to support the findings of this study are included within the article.
